# Voice Recognition and Evaluation of Vocal Music Based on Neural Network

**DOI:** 10.1155/2022/3466987

**Published:** 2022-05-20

**Authors:** Xiaochen Wang, Tao Wang

**Affiliations:** ^1^GuiZhou University of Finance and Economics, Guiyang, Guizhou 550000, China; ^2^Beijing Technology and Business University, Beijing 100048, China

## Abstract

Artistic voice is the artistic life of professional voice users. In the process of selecting and cultivating artistic performing talents, the evaluation of voice even occupies a very important position. Therefore, an appropriate evaluation of the artistic voice is crucial. With the development of art education, how to scientifically evaluate artistic voice training methods and fairly select artistic voice talents is an urgent need for objective evaluation of artistic voice. The current evaluation methods for artistic voices are time-consuming, laborious, and highly subjective. In the objective evaluation of artistic voice, the selection of evaluation acoustic parameters is very important. Attempt to extract the average energy, average frequency error, and average range error of singing voice by using speech analysis technology as the objective evaluation acoustic parameters, use neural network method to objectively evaluate the singing quality of artistic voice, and compare with the subjective evaluation of senior professional teachers. In this paper, voice analysis technology is used to extract the first formant, third formant, fundamental frequency, sound range, fundamental frequency perturbation, first formant perturbation, third formant perturbation, and average energy of singing acoustic parameters. By using BP neural network methods, the quality of singing was evaluated objectively and compared with the subjective evaluation of senior vocal professional teachers. The results show that the BP neural network method can accurately and objectively evaluate the quality of singing voice by using the evaluation parameters, which is helpful in scientifically guiding the selection and training of artistic voice talents.

## 1. Introduction

Artistic voice mainly refers to the singing voices appearing in artistic performances on the stage, movies, television, and radio, the singing voices, lines, and other animal voice shapes and voice effects in operas. It uses the color and style of the sound to create different images to express the content of the work and reflect the colorful life; it is efficient and subtle in sound modeling, versatile, and profound; it is the artistic life of professional voice users, and in the selection of in the process of cultivating artistic performance talents, the evaluation of voice even occupies a very important position. Therefore, an appropriate evaluation of the artistic voice is crucial [1–5].

Objective evaluation of artistic voice is an important part of medical research on artistic voice. Using microcomputer and acoustic knowledge to analyze artistic voice signal is an effective method to evaluate pronunciation. It has the advantages of noninvasiveness and objective and comparable data [6, 7]. Quantitative analysis and objective evaluation of various factors and laws in the pronunciation of singing artistic voices can help solve problems such as the selection of reasonable artistic voices, the evaluation and improvement of voice training methods, and the diagnosis and treatment of voice diseases.

At present, the most commonly used evaluation method in artistic voice evaluation is subjective listening perception evaluation, but the problems it faces cannot be ignored. For example, when selecting and cultivating artistic performance talents, the evaluation of vocal talents is basically based on the voice experts using their own experience to listen to and feel the sound quality of the test subjects as a whole and use simple scores or comments to represent the evaluation results. Due to the differences in the evaluation standards among the evaluators and the influence of various factors, the evaluation results are lacking in objectivity, accuracy, and fairness to a certain extent. Moreover, the results of subjective listening perception evaluation often cannot fully reflect the vocal condition of vocal talents, and it is difficult to provide an effective reference for various problems in vocal music teaching. Although some schools use voice medical examination as one of the reference basis for selecting artistic performing talents, the medical examination process will undoubtedly bring psychological and physical pain to candidates. In addition, since the evaluation of artistic voice runs through the whole process of talent selection, training, diagnosis, and treatment of voice problems, with the continuous increase of art students, the workload of voice evaluation has increased exponentially, thus affecting the human and material resources. Demand has also increased substantially, putting the evaluation of artistic voices in trouble. In order to solve the problems existing in the evaluation of subjective auditory perception, and to make the evaluation results more accurately reflect the functional state of people's voice during vocalization, it is necessary to find a new evaluation method, which takes the physical characteristics of the auditory as the standard and is not subject to subjective factors. With the rapid development of electronic technology and computer technology, the interaction between computers and other electronic products and human beings has become more and more extensive and in-depth [8–14]. They penetrate into almost every aspect of human life, give human beings great help, and also work for the voice. The speaker brought the gospel and made the objective evaluation of the artistic voice possible.

The objective evaluation of artistic voice not only plays a good guiding role in the scientific selection and training of singing and performing talents, but also plays a role in studying the vocal pathology of speakers and preventing and treating voice diseases. If you want the vocal music industry to become more and more prosperous, you must pay attention to the training and delivery of vocal talents. Singers, voice actors, performers, and vocal teachers need to protect their voices from further damage. Therefore, the correct objective evaluation of artistic voice is crucial. Researchers using computer and acoustics knowledge to explore objective and scientific evaluation methods for vocal quality in singing art have achieved initial results. Because of the noninvasive and excellent computing power of computers, its evaluation results are objective, reliable, accurate, and efficient. The purpose of objective evaluation of the voice includes the following aspects: (1) to increase the interest in singing; (2) to protect the tender voice; (3) to improve artistic accomplishment; (4) to evaluate the scope and extent of the disease; (5) to try to diagnose the disease; (6) after predicting and correcting the vocalization problem [15–20].

In the research of establishing the objective evaluation method of singing artistic voice, it is mainly divided into the evaluation method based on neural network and the evaluation method based on feature matching. The evaluation method based on neural network refers to the use of RBF network, BP neural network, CNN network, etc., to automatically extract discriminative features from the sound signal, and the use of softmax, support vector machine, and other classifiers to classify and discriminate the sound quality. It is a rating or score for an objective assessment of the quality of a singing voice. Neural networks have developed rapidly in recent years due to their excellent feature classification capabilities and the ability to stack multiple layers. Currently, the most advanced deep learning methods in the world are based on neural networks. Some people use the neural network method to build a model network for objective evaluation of artistic voices. The reasons for this are as follows: (1) from a probabilistic point of view, RBF does not have the same good probability characteristics as Softmax. (2) With the increase of the number of network layers, both the network structure and the complexity of the weight parameters that need to be trained increase accordingly, and the neural network has three prominent features such as local connection, weight sharing, and pooling operation, so the network structure is simple, the weight parameters are few, the training effect is good, and the classification accuracy rate is high. (3) The voice audio sample is an evaluation model of a one-dimensional signal neural network, which can reflect its characteristics more objectively. With the development of science and technology, the method of evaluating the quality of artistic voice based on artificial intelligence technology has been widely recognized by people in the vocal music industry. Therefore, it is theoretically and technically feasible to apply the neural network method to the objective evaluation of artistic voice in this paper [21–24].

To sum up, the objective evaluation of singing artistic voice is very meaningful for the selection and cultivation of singing artistic talents. It can not only select high-quality voices but also help improve the training methods of voices, so that singers can speak scientifically. More importantly, it allows singers to prevent related voice diseases, keep their voices young, and prolong their artistic life.

Therefore, using a computer to analyze the voice signal can effectively evaluate the quality of the sound quality, inability to carry out objective and fair evaluation of each voice sample and other defects. This paper analyzes the singing voice signal, extracts the characteristic parameters that characterize the singing voice, and uses the BP neural network to evaluate it objectively through machine learning and compare the evaluation results with the subjective evaluation [25, 26].

## 2. Acoustic Parameters

Singing is the language of art, the supplement and development of language. Artistic voice requires not only clear sentences, but also better sound quality. Because the core of this indicator is the voice, it is stipulated that the voice must be professional and artistic. A good artistic voice is characterized by penetrating singing, which can freely control the strength of breath and the level of energy. In addition, it should also have certain tension and endurance. The difference between an artistic voice and an ordinary voice is that the vocal cords of the former can freely control continuous vibration within a specified period of time, such as continuous vibration when singing. All in all, artistic voices exhibit many unique characteristics acoustically. Because acoustics is a discipline that studies the entire process of sound from generation, propagation to feedback, therefore, this is also the basis for studying scientific voices and screening qualified artistic voices.

The objective evaluation of singing is realized by computer programming in Matlab, and the first formant, third formant, fundamental frequency, sound range, fundamental frequency perturbation, first formant perturbation, third formant perturbation, and average energy of singing voice are extracted as evaluation parameters.

### 2.1. Formant Extraction

Formant is a theory that studies the resonance and quality of voice. In general, the lower two of these peaks, the first and second formants, basically define the vowel timbre of the sound, while the higher third, fourth, and fifth formants affect the personal character of the sound and the musical timbre. The long-term research results of domestic and foreign scholars on vocal formants in singing art show that the first and third formants are important objective reference data to measure the vocal technical level of singers. Therefore, the experiment selects the first and third formants as objective evaluation parameters and adopts the AR model peak detection method to extract the first and third formants. The formant time is plotted in Figure 1.

### 2.2. Fundamental Frequency Extraction

The fundamental frequency refers to the fundamental frequency at which the vocal cords vibrate, also known as the fundamental frequency. In addition to good timbre, an excellent artistic voice should also have a certain tension, that is, whether a certain sound can reach a certain height. Fundamental frequency is one of the important parameters for objective evaluation of artistic voice. There are many methods to extract fundamental frequency, such as autocorrelation function, average amplitude difference function, autocorrelation, and wavelet transform. After calculation and comparison, this experiment adopts the improved algorithm to extract the pitch period, so as to calculate the fundamental frequency. That is, the pitch period detection algorithm of artistic voice based on improved wavelet change mentioned later. The experimental steps are as follows:

1. Preprocess the original noisy signal, extract useful information segments from the processed signals, and combine these information segments into artistic voice segments.
2. Arrange the extracted artistic voice segments and filter out the DC components in them; then, set the signal-to-noise ratio to superimpose the noise; finally, use the DWT wavelet transform, and use the obtained low-frequency coefficients to reconstruct the target signal.
3. Perform pitch detection on the reconstructed artistic voice segment.

### 2.3. Sound Field Extraction Method

The simplest method for estimating the pitch range is to select the maximum and minimum pitch values that appear in the singing voice and musical score. However, there is much pitch data in the singing voice and musical score, and only two of them are selected, which is unavoidable by chance, and it is necessary to use statistical methods. The method of estimating the sound range in this experiment is to take the average and standard deviation of the *D* values of all pitches in the singing voice and score. The corrected autocorrelation waveforms before and after center clipping are compared in Figure 2.

Pitch is determined by the vibration frequency of the object (vocal cord). That is, if the number of vibrations in a certain unit time is large, the pitch will be high; if the number of vibrations is small, the sound will be low. Lin Tao and others pointed out in “Beijing Voice Experiment Record”: “Tone and intonation are both expressions of pitch. After all, pitch is not the direct reality of the fundamental frequency, but an abstraction cut across the pitch curve based on Hertz's things”. Therefore, the pitch is described by the *D* value in the experiment, which is the logarithmic scale of pitch and is defined as

(1) $$\begin{array}{c} D=12{}^{*}\;\log_{2}\left(\frac{F}{F_{0}}\right). \end{array}$$

That is, it is the step difference of the pitch *F* in Hertz with respect to the reference frequency *F*_0_. The *D* value is a dimensionless number, and its unit can be taken as “degree,” which is replaced by *D* for the convenience of writing.

Take the average and standard deviation of all pitch *D* values in the singing voice and score:

(2) $$\begin{array}{c} \bar{D}=\frac{1}{N}\sum_{j=1}^{N}D_{j}. \end{array}$$

The standard deviation *σ* is

(3) $$\begin{array}{c} \sigma =\sqrt{E\left[{\left(D_{j}-\bar{D}\right)}^{2}\right]}, \end{array}$$

where *E* represents the average, and *N* is the number of pitch data elements. The domain width S is

(4) $$\begin{array}{c} S=4\sigma . \end{array}$$

The fundamental frequency perturbation refers to the rate of change of the fundamental frequency of the sound wave between adjacent cycles, which is used to measure the difference between a specified cycle and the adjacent previous or next cycles, reflecting the frequency difference between the vocal cord vibration cycles. Mathematical definition of fundamental frequency perturbation:

(5) $$\begin{array}{c} Jitter=\frac{1}{N-1}\sum_{i=1}^{N}\left|\frac{1}{F_{0i}}-\frac{1}{F_{0\left(i-1\right)}}\right|. \end{array}$$

In the formula, *F* represents the fundamental frequency of the ith cycle.

The first and third formant perturbations measure the rate of change of the first and third formants between adjacent periods, respectively. The mathematical definitions of formant perturbation are as follows:

(6) $$\begin{array}{c} \frac{1}{N-1}\sum_{i=1}^{N}\left|\frac{1}{F_{1i}}-\frac{1}{F_{1\left(i-1\right)}}\right|,\\ \frac{1}{N-1}\sum_{i=1}^{N}\left|\frac{1}{F_{3i}}-\frac{1}{F_{3\left(i-1\right)}}\right|. \end{array}$$

The average energy represents the relative magnitude of the singing voice signal in the same environment. Mathematical definition of short-term energy of speech signal:

(7) $$\begin{array}{c} E_{n}=\sum_{k=-\infty }^{+\infty }x^{2}\left(k\right)w\left(n-k\right). \end{array}$$

## 3. Neural Networks

Since the neural network is formed by imitating the biological neural network of the human brain, it is very close to the operating rules of the human brain when processing information and has strong self-learning and adaptive capabilities. The network automatically adjusts its structure according to different input samples. Parameters to give the desired output: because the knowledge is stored in the connection weights, the neural network can realize various nonlinear mappings by adjusting the weights; due to the relative independence between neurons in each layer, when the neural network stores information, it is distributed, so its robustness and fault tolerance are good; in addition, the neural network is composed of a large number of simple processing units connected in parallel, making it extremely easy to implement in hardware and running extremely fast.

These characteristics of neural network make it have a very good performance in many fields, and it has played an important role in many industries such as aerospace, automotive, manufacturing, finance, and telecommunications. The characteristics of neural network make it especially suitable for speech signal processing. Since 1980, the application of neural network in speech signal processing has been very active, and the more prominent one is speech recognition. This paper attempts to use the neural network method to evaluate the level of artistic voice signals.

A neural network is an information processing system or mathematical model that imitates the function of the human brain, and there are many different network models. Since the objective evaluation of singing needs to determine the weights (weight coefficients) of each evaluation parameter, the backpropagation network model, often called the BP network model, is selected. Through the reverse adjustment of the weights in the network learning process, each weight can be obtained, a set of optimal solutions. BP neural network includes input layer, hidden layer, and output layer. Using BP neural network to objectively evaluate singing includes two processes, training process and evaluation process, the training process is based on the evaluation parameters of the training samples and the corresponding subjective evaluation scores through neural network learning and training to establish an evaluation model; the evaluation process uses the evaluation parameters of the samples to be evaluated. Input the established evaluation model, get the objective evaluation score, and compare it with the corresponding subjective evaluation score to test the usability of the established evaluation model (see Figure 3).

The BP neural network adopts the error back propagation learning algorithm, which is based on the Delta learning rule and uses the gradient search technology to minimize the mean square error between the actual output and the expected output of the network. The process of network learning is a process of correcting weights while propagating backwards. In such a network, the learning process consists of forward propagation and backpropagation. In the forward process, the input signal is processed layer by layer from the input layer through the hidden layer unit and transmitted to the output layer. The state of each layer of neurons only affects the state of the next layer of neurons. If the expected output cannot be obtained at the output layer, turn to backpropagation and return the output error according to the original connection path. By modifying the weights of neurons in each layer, the error signal is minimized. Once the appropriate network connection values are obtained, the new samples can be nonlinearly mapped.

Use *S*_*j*_ to calculate the output *b*_*j*_ of each intermediate unit through the transfer function:

(8) $$\begin{array}{c} S_{j}=\sum_{i=1}^{n}w_{ij}a_{i}-\theta_{j},\\ b_{j}=f\left(s_{j}\right). \end{array}$$

Use the output *b*_*j*_ of the intermediate layer, the connection weight *v*_*jt*_ and the threshold *γ* to calculate the output *L*_*t*_ of each unit of the output layer, and then use the transfer function to calculate the response *C*_*t*_ of each unit of the output layer.

(9) $$\begin{array}{c} L_{t}=\sum_{j=1}^{p}v_{jt}b_{j}-\gamma_{t},\\ C_{t}=f\left(L_{t}\right). \end{array}$$

Theoretically, it has been shown that a network with bias and at least one sigmoid hidden layer plus a linear output layer can approximate any rational number. Increasing the number of layers can further reduce the error and improve the accuracy, but it also complicates the network, thereby increasing the training time of the network weights. The improvement of error accuracy can actually be obtained by increasing the number of neurons, and its training effect is easier to observe and adjust than increasing the number of layers. In general, priority should be given to increasing the number of neurons in the hidden layer.

The improvement of network training accuracy can be obtained by using a hidden layer and increasing the number of neurons. In terms of structure implementation, it is much simpler than increasing the number of hidden layers. How many hidden layer nodes to select is appropriate, and there is no clear regulation in theory. In the specific design, the more practical way is to compare the training of different numbers of neurons and then add a little margin appropriately. More broadly, the number of neurons in the hidden layer = 2 *∗* the number of input layers: 4 *∗* the number of input layers. Since the system is nonlinear, the initial value is very important to whether the learning reaches a local minimum, whether it can converge, and the length of the training time. If the initial value is too large, the weighted input sum *n* falls into the saturation region of the s-shaped activation function, causing its derivative to be very small, which makes the revised weights close to zero, and the adjustment process almost stops. Therefore, it is generally hoped that the output value of each neuron after initial weighting is close to zero, which ensures that the weights of each neuron can be adjusted where their sigmoid activation function changes the most. Therefore, a random number with an initial weight between (−1, l) is generally taken.

The learning rate determines the amount of weight change produced in each loop training. A large learning rate may lead to instability of the system; but a small learning rate leads to a longer training time and may converge very slowly, but it can ensure that the error value of the network will not jump out of the trough of the error surface and eventually tend to the minimum error value. Therefore, in general, we tend to choose a smaller learning rate to ensure the stability of the system. The learning rate is selected in the range of 0.01–0.8. The prediction comparison is shown in Figure 4.

## 4. Simulation Experiments

Although subjective auditory perception evaluation is affected by subjective factors and has problems such as low accuracy and stability, it is undeniable that subjective auditory perception evaluation is the only reference standard for testing and evaluating the effectiveness of objective test parameters of voice and vocal function inspection. In order to provide a supervisory signal to the input training samples of the neural network and verify the effectiveness of the objective evaluation method in this paper, this paper conducts subjective listening perception evaluation of artistic voice signal. In order to verify the practicability of the objective evaluation method in this paper, two vocal music teachers and two vocal music graduate students were invited as judges to listen to 22 singing recording materials separately and scored on a 10-point scale, and the average score was taken, and the score was greater than 6 points. A score of less than 6 is considered poor. Put the subjective evaluation results together with the fundamental frequency, F1, F3, extracted from the corresponding samples to prepare for the experiment.

The objective evaluation process includes training process and evaluation process. In the training process, the evaluation parameters of the training samples and their subjective evaluation results are learned through a neural network to obtain a trained network; in the evaluation process, the evaluation parameters of the remaining samples to be tested are input into the trained network to obtain objective evaluation results. The objective evaluation results were compared with the corresponding subjective evaluation results to test the accuracy of the neural network artistic voice objective evaluation model after training on the voice evaluation results. Neural network is a nonlinear system, which can fully approximate nonlinear systems of arbitrary complexity and has the ability of self-organization, self-adaptation, and self-learning for information processing. Error Backpropagation (BP) neural network is a multilayer feedforward neural network with continuous transfer function. The training method is the error backpropagation algorithm, and the weights and thresholds of the network are constantly modified with the goal of minimizing the mean square error. Finally, the high-precision fitting of the data is carried out. In this paper, the BP neural network is used to objectively evaluate the artistic voice. The objective evaluation process of artistic voice includes training process and evaluation process. The training process will randomly select the evaluation parameters of the training samples and their subjective evaluation results through the BP neural network to learn to obtain the trained network; the evaluation process will input the evaluation parameters of the remaining samples to be tested into the trained network to obtain the objective evaluation results, which are combined with the results. The corresponding subjective evaluation results are compared to test the correctness of the voice evaluation results of the trained BP neural network. The error is plotted in Figure 5.

The specific process selects the first formant, the third formant, the fundamental frequency, the pitch range, the fundamental frequency perturbation, the first formant perturbation, the third formant perturbation, and the average energy of the training sample singing voice as evaluation parameters and normalizes and eliminates the effects of different orders of magnitude that are used as input parameters, and the scores scored by senior professional teachers in subjective evaluation of singing quality are used as output parameters to establish a nonlinear relationship model between training sample singing quality scores and evaluation parameters. After repeating the training, it is found that the neural network with the number of neurons in the hidden layer of 25 has the smallest approximation error to the singing training samples, so the number of neurons in the hidden layer is selected as 25, and the transfer functions of the hidden layer and the output layer are selected as tansig and logsig, respectively. The initial values of the weights and thresholds are random numbers between [0, 1], and the maximum training error is set to 0.001. The optimal connection weights and thresholds are obtained through the training and learning of the neural network, and the neural network evaluation model is obtained. Finally, the parameters of the singing voice samples to be evaluated are used as input parameters, and the score of the singing voice is predicted by the trained neural network model.

Figure 6 shows the differences between the objective evaluation scores and the subjective evaluation scores. Comparing the error between the objective evaluation scores and the subjective evaluation scores of senior professional teachers, the neural network method is within 3.4%. Since the number of high scores and low scores in the singing samples is small, and this is also the case for the randomly selected training set, the error between high scores and low scores is relatively large in objective evaluation.

Randomly select 6 good and bad singing signals from the subjective evaluation results, as the input of training samples, and get the trained network after training. Input the remaining 10 singing samples to be tested into the trained network to obtain objective evaluation results. When the final iteration number is 2000, the mean square error between the expected output and the actual output is calculated to be 0.1891, as shown in Figure 7. At this time, compared with subjective evaluation, the correct rate of objective evaluation reaches 90%. The distribution of the 12 samples involved in training is shown in Figure 8.

From the perspective of data normalization, since the BP neural network uses the idea of gradient descent to adjust the parameters of the network, the range of the input data will affect the update of the gradient value, influencing and improving the accuracy of the network evaluation results, and the input acoustic parameters need to be normalized, so the training time of the BP neural network is relatively long; the improved neural network is developed from the associative learning theory and competitive algorithms. As long as the distance between the input vector and the competition layer is directly calculated, there is no need to normalize and orthogonalize the data, so it is simpler and easier to realize the objective evaluation of artistic voice.

From the perspective of network training, the choice of the number of neurons in the hidden layer/competitive layer has a great impact on the performance of the network. Generally, a larger number of neurons in the hidden layer/competitive layer can bring better performance. However, the network structure will be more complex, resulting in too long training time. In the training of the BP neural network, the number of neurons in the hidden layer is selected to be 14 to obtain the smallest training error, while the number of neurons in the competition layer of the improved neural network is set to 7. The minimum training error can be achieved. The number of training steps also affects the training time of the network. The more the training steps, the longer the training time. Experiments show that when the training errors of the BP neural network and the improved neural network reach the minimum, the training time is 10 seconds and 8 seconds, respectively. From the evaluation results, the use of BP neural network and improved neural network to objectively evaluate artistic voice signals can achieve satisfactory results. The accuracy of the BP method is 85.2%, and the accuracy of the improved method is 88.9%.

## 5. Conclusion

In this paper, the first formant, the third formant, the fundamental frequency, the pitch range, the fundamental frequency perturbation, the first formant perturbation, the third formant perturbation, and the average energy of the singing sample are extracted by speech analysis technology as evaluation parameters. The network method objectively evaluates the singing quality, and the results show that the objective evaluation is consistent with the subjective evaluation of senior professional teachers. Because artistic voice singing is affected by multiple factors, and there is a complex mutual influence relationship between each factor, it has a highly uncertain nonlinear relationship. The neural network method considers the nonlinear mapping relationship between them and evaluates the singing voice. The quality is accurate. The experimental results show that the multiparameter artistic voice objective evaluation model established by the training samples has good consistency with the subjective auditory evaluation results and can comprehensively reflect the physiological function of the larynx.

Based on the above experimental results, the objective evaluation of singing artistic voice needs to be further improved and developed as follows: gender, vocal part increases male bass, middle, soprano and female bass, and middle and soprano singers. The evaluation model is established by gender, so as to more comprehensively explore the quantitative impact of various acoustic characteristic parameters on the sound quality, so as to allow singers to better grasp the vocalization laws and characteristics, and to more scientifically adjust the use of each vocalization organ.

## Figures and Tables

**Figure 1:** Formant time plot.

**Figure 2:** Corrected autocorrelation waveforms before and after center clipping.

**Figure 3:** The established evaluation model.

**Figure 4:** Prediction comparison.

**Figure 5:** Error.

**Figure 6:** Differences between the objective evaluation and the subjective evaluation.

**Figure 7:** Convergence.

**Figure 8:** Evaluated value.

## Data Availability

The dataset can be accessed upon request.
